This article has been retracted.

# Inhibition Effect of Zoledronate on the Osteoclast Differentiation of RAW264.7 Induced by Titanium Particles

**DOI:** 10.1155/2021/5578088

**Published:** 2021-03-04

**Authors:** Wenhan Zhao, Zhusong Huang, Yu Lin, Jinfu Lan, Xi Gao

**Affiliations:** Department of Orthopaedics, Fuzhou Second Hospital affiliated to Xiamen University, Fujian Province 350007, China

## Abstract

**Objective:**

This study is aimed at studying the effect of zoledronate (ZOL) on the differentiation of osteoclast precursor RAW264.7 cells induced by titanium (Ti) particles and explores the possibility of preventing and treating periprosthetic osteoporosis using ZOL.

**Methods:**

RAW264.7 cells were cultured in vitro. Ti particles were prepared. The cell proliferation curve of RAW264.7 cells was plotted using the MTT assay to find the best concentration of ZOL for intervention. The cells were divided into three groups: control, Ti particles, and Ti particles+ZOL. The cell morphology was observed using tartaric acid–resistant acid phosphatase (TRAP) staining, and the activity of TRAP in cell supernatant was determined using the biochemical method. The number of bone resorption lacunae was detected using toluidine blue staining. The mRNA expression of *RANK*, *NFATcl*, *CAII*, and *MMP-9* was detected using real-time polymerase chain reaction. The protein expression of RANK, NFATcl, and MMP-9 was detected using Western blot analysis.

**Results:**

Ti particles stimulated the differentiation of RAW264.7 cells into osteoclasts. They also increased the activity of TRAP, number of bone resorption lacunae, and mRNA and protein expression of RANK, NFATcl, and MMP-9. However, ZOL could suppress the effect of TI particles on the osteoclast differentiation of RAW264.7 cells.

**Conclusions:**

ZOL could effectively inhibit the differentiation of RAW264.7 cells into osteoclasts induced by Ti particles, decrease the activity of TRAP, reduce the number of bone resorption lacunae, and decrease the mRNA and protein expression of RANK, NFATcl, and MMP-9. Hence, it may be a promising candidate for preventing and treating periprosthetic osteoporosis after the artificial joint operation.

## 1. Introduction

The number of hip fractures caused by trauma, osteonecrosis of the femoral head, and osteoporosis has increased with the aging of the population in China. Total hip arthroplasty (THA) has become the main way to restore the hip function [1]. However, the aseptic loosening of the prosthesis caused by periprosthetic osteoporosis after THA operation is the main factor affecting the stability of the hip joint, the service life of the prosthesis, and the renovation rate [2]. The osteoclast precursor cells have been found to gather around the foreign body and differentiate into osteoclasts, which indicates their important role in periprosthetic osteoporosis. With the excellent mechanical strength and biocompatibility, titanium (Ti) particles have been widely used for fabrication of prosthesis in THA [3]. Previous studies demonstrated that the metal and polyethylene liner produced a large number of metal particles and subparticles due to continuous wear after replacement, and the shed particles moved to the bone–prosthesis interface with mechanical fretting. These prosthetic wear particles, such as Ti particles, have been reportedly involved in the initiation and development of periprosthetic osteoporosis by promoting osteoclast differentiation and bone resorption activity [4, 5]. The formation of debris particles on the prosthesis is unavoidable; although, surgical techniques, prosthetic materials, and manufacturing techniques have been significantly improved. Thus, identification of drugs that can inhibit the activation of osteoclasts caused by debris particles to minimize the production of debris particles is important to solve the loosening of the prosthesis caused by periprosthetic osteoporosis.

Bisphosphonates (BPs) are a major class of pyrophosphate analogues that have been used for treating several skeletal-related diseases, such as osteoporosis and bone metastases. Their therapeutical effects mainly depend on the antiosteoclastogenic effect and inhibitory action on bone resorption by being selectively taken up to mineral surfaces in the bone [6]. Zoledronate (ZOL), one of the nitrogen-containing BPs (N-BPs), has been widely used for treating osteoporosis [7, 8]. It can increase the periprosthetic bone mass by inhibiting the differentiation of osteoclasts around the prosthesis and slowing down the rate of bone reconstruction [9, 10]. It has been shown that ZOL can inhibit RANKL-induced osteoclast differentiation by targeted suppression of NFATc1 and CAII gene expression [11]. And ZOL can enhance osteocyte-mediated osteoclastogenesis through the elevated expression of IL-6, the sclerostin mRNA, and subsequent RANKL expression [12], but its effects on osteoclast precursor cells and the activation of osteoclasts still remain to be found. Therefore, this study was conducted to investigate the effect of ZOL intervention on the differentiation of osteoclast precursor RAW264.7 cells induced by Ti particles so as to provide evidence for the clinical application of ZOL to prevent aseptic loosening caused by periprosthetic osteoporosis after THA.

## 2. Materials and Methods

### 2.1. Experimental Materials

#### 2.1.1. Drugs and Cells

ZOL was supplied by Beijing Novartis Pharmaceutical Co., Ltd., China (size: 5 mg/100 mL, import drug registration No. H20070127). RAW264.7 mouse mononuclear macrophage leukemia cells were purchased from Guangzhou Ginio Biotechnology Co., Ltd., China.

#### 2.1.2. Main Reagents and Test Instruments

The Ti particles with an average diameter of 0.91 ± 0.65 *μ*m were provided by the Beijing Nonferrous Metals Company. Tartrate-resistant acid phosphatase staining kit was procured from Nanjing Institute of Biological Engineering, China. TRIzol was bought from Invitrogen. PrimeScript reverse transcription reagent kit and SYBR Green Premix Ex Taq Polymerase Chain Reaction (PCR) Kit were purchased from TaKaRa; PCR primers were procured from Shanghai Bioengineering Technology & Technology Co., Ltd., China. Antibodies against RANK, NFATcl, MMP-9, and *β*-actin were obtained from Cell Signaling. ELx800 enzyme-labeled meter was purchased from Bio-Tek. The PCR amplification system 9600 was procured from the PE Company (USA). The 7500 Fast real-time quantitative PCR instrument was purchased from the ABI Company (USA). The polychromatic fluorescence/chemiluminescence imaging system was obtained from the ProteinSimple Company (USA).

### 2.2. Experimental Method

#### 2.2.1. Pretreatment of Ti Particles before Intervention

First, the Ti particles were placed in the oven at 300°C for 6 h. The Ti particles (100 mg) were suspended in 25 mL of 75% ethanol to make the suspension. The particle suspension was put on a horizontal rocker with a speed of 200 rpm, and the supernatant was removed by centrifugation after 24 h. Then, the sample was replaced with ethanol and oscillated for 24 h. The liquid was removed by centrifugation and washed three times. After drying again, it was exposed to ultraviolet for 24 h. The concentration of endotoxin in Ti particles after treatment was measured: if the concentration was less than 0.10 EUP/mL, the effect of endotoxin on cells could be excluded. Finally, the pretreated Ti particles were placed in DPBS, and the volume ratio of 0.1% (v/v) of suspension was prepared, in which 1 mL finally contained 4.5 × 10^7^ Ti particles. Before intervention, 10 min oscillation was conducted using an ultrasonic magnetic oscillator to eliminate adhesions.

#### 2.2.2. Effect of ZOL on the Proliferation of RAW264.7 Cells

RAW264.7 cells were plated in a 96-well culture plate. The old culture medium was abandoned overnight, and the cells with concentrations of 0 mol/L, 10^–9^ mol/L, 10^–8^ mol/L, 10^–7^ mol/L, 10^–6^ mol/L, 10^–5^ mol/L, 10^–4^mol/L, 10^–3^mol/L, 10^–2^mol/L, and 10^–1^ mol/L were added to the cell culture plate containing ZOL. Eight wells were set for each concentration of cells. After culturing for 72 h, the cells were treated with 20 *μ*L of tetrazolium salt solution (5 g/L) for each well. The supernatant was removed after incubation for 4 h at 37°C. After adding 150 *μ*L of DMSO in each well, the cell samples were oscillated on the rocking bed for 10 min. The absorbance value of each well was measured using the enzyme-labeled meter by selecting a 490 nm wavelength, and its value was proportional to the number of cells.

#### 2.2.3. Coculture of RAW264.7 Cells with Ti Particles and ZOL Intervention

RAW264.7 cells were plated on a six-well plate at a concentration of 1 × 10^6^/well and placed in the incubator overnight. They were divided into three groups: control (conventional medium containing 10% fetal bovine serum), Ti particles (medium containing 0.1% volume of Ti particles and 10% fetal bovine serum), and Ti+ZOL (medium containing 0.1% volume of Ti particles, 10% fetal bovine serum, and optimum concentration of ZOL). The cells were cultured continuously for 48 h after intervention. The differentiation of RAW264.7 cells into osteoclasts was observed using TRAP staining.

#### 2.2.4. Detection of TRAP Activity in Cell Suspension Using the Biochemical Method

After the 48-h intervention, the cell culture medium was added to the test tube. Triton X-100 (0.2%; 0.05 mL for each tube) was used for cell lysis. Distilled water (0.05 mL) and 0.1 mg/mL phenol standard application solution were added to the empty test tube, and then 0.5 mL of buffer solution and 0.5 mL of substrate solution were added. After fully mixing, the mixture was incubated at 37°C for 15 min. Finally, 1.5 mL of chromogenic agent was added. After immediate mixing, the absorbance of each tube was measured at a wavelength of 520 nm using 0.5 cm diameter colorimeter with blank tube zero adjustment.

#### 2.2.5. Observation of Cortical Bone Resorption Lacunae Using Toluidine Blue Staining

The cortical bone was pruned to the size of 0.5 × 0.5 cm^2^, ultrasonically cleaned with ultrapure water three times, and soaked in 75% ethanol for 2 h. It was irradiated using an ultraviolet lamp in the ultra-clean worktable for 1 h and then soaked in the high-sugar DMEM medium for 1 h. A 24-well plate was used. One piece of bone mill was placed in each well and mixed with Ti particles in the Ti particles and Ti + ZOL groups with a density of Ti particles of 2 × 10^3^/well. The bone mill was taken out on the 10th day of coculture in the Ti particles and Ti+ZOL groups. The sample was fixed, dehydrated using gradient ethanol, dried, stained with 0.5% toluidine blue dye, and washed with water. Finally, the bone resorption pit was observed under a microscope.

#### 2.2.6. Detection of the mRNA Expression of RANK, NFATcl, CAII, and MMP-9 Using Real-Time qPCR (RT-qPCR)

Total RNA of cells was extracted using the TRIzol method, and the ratio of A260/A280 was calculated to obtain the concentration of RNA. Then, 500 ng RNA was used to synthesize cDNA using a reverse transcription kit, and the cDNA was stored at 20°C for real-time fluorescence quantification on ABI 7500 Fast PCR machine. The primers used are shown in Table 1. CT values, the expanded curve, and the dissolution curve were obtained after 40 cycles of PCR using 20 *μ*L of the SYBR Green reaction system. Three multiple holes for each index were set for each sample. The CT values obtained were converted into the relative expression of the target gene using the 2^-*ΔΔ*Ct^ method.

#### 2.2.7. Detection of the Protein Expression of RANK, NFATcl, and MMP-9 Using Western Blot Analysis

The cell scraper was employed to collect the cells. The total protein was extracted, and the protein concentration was measured using the bicinchoninic method. Each lane was loaded with 30 *μ*g of protein, and 12% sodium dodecyl sulfate–polyacrylamide gel electrophoresis was conducted. The proteins were transferred to the polyvinylidene difluoride membrane using the half-dry method, and the blocking solution was used to incubate with the proteins at room temperature for 30 min. The rinsing membrane was washed six times after incubation with the primary antibody at room temperature for 1 h. Then, the secondary antibody was added and incubated with the proteins at room temperature for 30 min, and the membrane was washed five times. The chemiluminescence substrate AP was incubated with the membrane at room temperature for 5 min. The film was exposed and developed. The Phoretix 1D bioelectrophoretic image analysis system was used to analyze the bands of proteins in the film. The optical density of each band was automatically read and recorded using a computer.

#### 2.2.8. Statistical Analysis

The data were analyzed using SPSS18.0 software, and the measurement data were expressed as mean ± standard deviation (SD). The normality of the test data and the homogeneity of variance were tested. The *F* test and then the *Q* test were used for comparison among the groups. A *P* value less than 0.05 indicated a statistically significant difference between the two groups.

## 3. Results

### 3.1. Effect of ZOL on the Proliferation of RAW264.7 Cells

The effects of different concentrations of ZOL on the proliferation of RAW264.7 cells were compared, and the optimum concentration of intervention was determined. The RAW264.7 cell proliferation curve was plotted using the MTT method. The results showed no obvious change for ZOL concentration range of 0–10^−6^ mol/L. Then, the cell proliferation ability decreased gradually with the increase in ZOL concentration. Therefore, 10^−6^ mol/L ZOL was determined as the best concentration of intervention in this study (Figure 1).

### 3.2. ZOL Decreases Osteoclast Differentiation of RAW264.7 Cells Induced by Ti Particles

The microscopic observation revealed that the number of RAW264.7 cell nuclei and pseudopodia increased after coculture with Ti particles, and the cells were not arranged evenly. The cells were treated with TRAP staining after the treatment of RAW264.7 cells with Ti particles with or without ZOL. A brown-red precipitate was formed in the cytoplasm of cells, and the nuclei were stained negative. The Ti particles group had the most obvious change, followed by the Ti + ZOL group, while the control group had no obvious change (Figure 2). These results suggested that ZOL suppressed Ti particle-induced osteoclastogenesis.

### 3.3. ZOL Inhibits the Number of Bone Resorption Lacunae in RAW264.7 Cells Induced by Ti Particles

The number of bone resorption lacunae in the Ti particle group significantly increased (*P* < 0.01), and the size of the lacunae was not uniform. The number of bone resorption lacunae in the Ti + ZOL group decreased, and occasionally, larger bone resorption lacunae were found (*P* < 0.01) (Figures 3(a) and 3(b)).

### 3.4. ZOL Suppresses Ti Particle-Induced Osteoclast-Associated Gene Expression

The expression of osteoclast-related gene RANK, NFATcl, CAII, and MMP-9 was detected. The mRNA expressions of RANK, NFATcl, CAII, and MMP-9 significantly increased in the Ti particle and Ti + ZOL groups compared with the control group (*P* < 0.05). The mRNA expression of RANK, NFATcl, CAII, and MMP-9 decreased to a certain extent compared with the Ti particle group (*P* < 0.05), with a significant difference between the two groups (*P* < 0.05) (Figure 4).

Furthermore, the protein expression of RANK, NFATcl, and MMP-9 significantly increased in the Ti particle group compared with the control group (*P* < 0.01). The protein expression of RANK, NFATcl, and MMP-9 decreased to some extent (*P* < 0.01) compared with the Ti particle group. A significant difference was found between groups (Figure 5).

## 4. Discussion

THA is an ideal method for treating advanced hip joint disease. The long-term survival rate of prosthesis is mainly affected by prosthesis loosening, with a significant relationship between prosthesis loosening and loss of bone mass around prosthesis [13, 14]. After the implantation of THA prosthesis, the wear particles around the prosthesis have a chemotactic effect on monocytes, recruiting the monocytes around the prosthesis. Therefore, inhibiting the activation of osteoclasts, prolonging the prosthesis service life, and reducing the rate of joint revision, besides improving the prosthetic material and manufacturing process of the prosthesis to minimize the production of debris particles and improve the surgical techniques, are important to solve the loosening of the prosthesis caused by periprosthetic osteoporosis.

In the present study, Ti particles significantly increased the activity of TRAP, number of bone resorption lacunae, and the expression of RANK, NFATcl, and MMP-9 in RAW264.7 cells. RANK is located on osteoclast precursor cells and can be recognized by RANKL. The formation and activation of osteoclasts are induced after RANK binds to the osteoclast receptor [15, 16]. NFATcl is the most important factor in the process of osteoclast differentiation mediated by RANKL, which can activate the downstream RANKL/RANK pathway, promote the differentiation of osteoclast precursor cells RAW264.7 into osteoclasts [17, 18], and induce the expression of various specific genes in osteoclasts, such as TRAP and CAII [19]. TRAP mainly exists in macrophages, osteoclasts, and mononuclear phagocytes. It is an important enzyme and histochemical identification marker of osteoclasts [20, 21]. MMP-9 is specifically and highly expressed in osteoclasts. It can specifically degrade nonmineralized cartilage and release vascular endothelial growth factor combined with the extracellular matrix. It causes direct chemotaxis and activation of osteoclasts. At the same time, it also has an important role in the migration of osteoclasts to the bone surface [22, 23]. Thus, our results suggested that Ti particles could promote the transformation of monocytes into osteoclasts.

ZOL is the newest preparation of bisphosphates. It can inhibit osteolysis caused by the activation of the osteoclast function by debris particles of prosthesis and improve the biological fixation effect of the prosthesis through close binding of the heterocyclic ring of diazoimidazole with the bone [24]. Previous studies showed that ZOL could inhibit the periprosthetic osteolysis of the aseptic loosening dog model after THA operation, improve the biomechanical properties of the cortical bone by increasing the bone density of periprosthesis, and protect the intramembranous ossification [25, 26]. In addition, ZOL inhibited the isoprene synthesis associated with the structure of osteoclasts through inhibition of phenyl pyrophosphate synthase by blocking the metabolic pathway of mevalonic acid [27, 28]. It also inhibited the expression of integrin *α*_v_ and *β*_3_ in osteoclasts. Thus, the role of osteoclasts in adhesion, cytoskeleton rearrangement, and bone resorption was affected [29]. Moreover, apoptosis of osteoclast precursors and mature osteoclast-like cells was induced by triggering the reactive oxygen species and glycogen synthase kinase-3 (GSK-3) [30]. In this study, after the intervention of ZOL, the expression of RANK, NFATcl, CAII, MMP-9, and the TRAP activity significantly decreased in the Ti particle group. It indicated that ZOL might block the binding of RANK receptor, inhibit the expression of NFATcl, and downregulate the expression of TRAP and MMP-9 in RAW264.7 cells through the RANKL/RANK pathway, which ultimately inhibited the differentiation and maturation of osteoclasts and thus reduced the bone resorption function of osteoclasts.

## 5. Conclusion

In conclusion, ZOL could inhibit the differentiation of RAW264.7 cells into osteoclasts induced by Ti particles. However, the long-term effect of ZOL on bone resorption around joint prosthesis and the inhibitory effect on inflammatory factors produced by debris particles on prosthesis need further investigation in vivo.

## Figures and Tables

**Figure 1:** Effects of different concentrations of ZOL on the proliferation of RAW264.7 cells. RAW264.7 cells were treated with different concentrations of ZOL (0, 10^–9^, 10^–8^, 10^–7^, 10^–6^, 10^–5^, 10^–4^, 10^–3^, 10^–2^, and 10^–1^ mol/L), and cell proliferation was detected by MTT after 72 h. ZOL: zoledronate.

**Figure 2:** Effect of ZOL on TRAP staining of RAW264.7 cells induced by Ti particles. RAW264.7 cells were cultured with Ti particles in the presence or absence of ZOL (10^−6^ mol/L) for 48 h and then stained with TRAP (magnification ×100). ^∗∗^*P* < 0.01 vs. control group; ^##^*P* < 0.01 vs. Ti group.

**Figure 3:** ZOL inhibits the number of bone resorption lacunae in RAW264.7 cells induced by Ti particles. RAW264.7 cells were cultured with Ti particles in the presence or absence of ZOL (10^−6^ mol/L) and then stained with Toluidine blue staining (100×) (a). (b) Quantitative analysis of number of bone resorption lacunae. ^∗∗^*P* < 0.01 vs. Ti group.

**Figure 4:** ZOL inhibits Ti particle-induced osteoclast-associated gene expression. The mRNA expression of osteoclast-associated genes was measured by RT-qPCR. ^∗∗^*P* < 0.01 vs. control group; ^##^*P* < 0.01 vs. Ti group.

**Figure 5:** ZOL inhibits Ti particle-induced osteoclast-associated protein expression. The protein expression of osteoclast-specific genes was detected by Western blot. ^∗∗^*P* < 0.01 vs. control group; ^##^*P* < 0.01 vs. Ti group.

**Table 1:** Primer sequences of real-time PCR.

Genes	Forward primers (5′-3′)	Reverse primers (5′-3′)
RANK	TCATCGTTCTGCTCCTCTTCA	CATCTTCTCCTCCCGAGTCAT
NFATcl	CAAGTCTCACCACAGGGCTCACTA	TCAGCCGTCCCAATGAACAG
CAII	AGGGAGGCCCATTACTACG	ATTCCAAATCACCCAGCGCGT
MMP-9	CCTCCGTTGTCCTGTAAATCTGC	TCTGACGCTGAAACCATAACGCA
GAPDH	CCGAAATGGGAAGCTTGTC	AAGCACCAGAGAGGAGAA

## Data Availability

Some or all data, models, or code generated or used during the study are available from the corresponding author by request.
